The article "Protective effects of fruit extract of Rosa canina and quercetin on human umbilical vein endothelial cell injury induced by hydrogen peroxide" was retracted in 2025. Reasons: errors in the analysis; unreliable results or conclusions; concerns about the images.

# Protective effects of fruit extract of *Rosa canina* and quercetin on human umbilical vein endothelial cell injury induced by hydrogen peroxide

**DOI:** 10.1002/fsn3.3681

**Published:** 2023-09-28

**Authors:** Fatemeh Forouzanfar, Zeynab Tabatabaei, Seyed Ahmad Emami, Zahra Ayati, Zahra Tayarani‐Najaran

**Affiliations:** ^1^ Department of Neuroscience, Faculty of Medicine Mashhad University of Medical Sciences Mashhad Iran; ^2^ Department of Traditional Pharmacy, School of Pharmacy Mashhad University of Medical Sciences Mashhad Iran; ^3^ Western Sydney University Penrith Australia; ^4^ Targeted Drug Delivery Research Center, Pharmaceutical Technology Institute Mashhad University of Medical Sciences Mashhad Iran; ^5^ Medical Toxicology Research Center Mashhad University of Medical Sciences Mashhad Iran

**Keywords:** apoptosis, cardiovascular diseases, cytoprotection, oxidative damage, quercetin, *Rosa canina*

## Abstract

The Nastaran plant, with the scientific name of *Rosa canina*, has been used since ancient times as a plant with medicinal properties. In the present study, human umbilical vein endothelial cells (HUVECs) were used to examine the protective effects of *R. canina* fruit extract (RCFE) and its flavonoid ingredient (quercetin) against H_2_O_2_‐induced cell injury. RCFE (1.25–20 μg/mL) and quercetin (1.25–20 μM) were exposed to H_2_O_2_‐oxidizing agent (1 and 2 mM) and the protective effect was examined on HUVEC cells by Alamar Blue test. The amount of intracellular reactive oxygen species (ROS) was measured by using DCFDA reagent by fluorimetric method. The effects of RCFE and quercetin on cell apoptosis were studied by staining with hypotonic PI solution and flow cytometry. The amount of PARP and survivin involved in the apoptotic process was measured using the western blot analysis. The results of the Alamar Blue test showed that RCFE and quercetin could reduce the toxicity of H_2_O_2_. RCFE and quercetin were able to significantly increase cell viability against H_2_O_2_. Also, it was found that RCFE and quercetin reduced the production of ROS by H_2_O_2_. It was found that RCFE and quercetin reduced the apoptosis and sub‐G1 peak area in flow histogram after exposure of cells to H_2_O_2_. Based on western blot results, pretreatment with RCFE and quercetin could significantly increase survivin protein after exposure of cells to H_2_O_2_. Also, RCFE and quercetin could significantly reduce the amount of cleaved PARP after exposure of cells to H_2_O_2_. RCFE and its ingredient (quercetin) can be considered a promising source of phytochemicals in the prevention of cardiovascular diseases.

## Graphical abstract

*Rosa canina* extract and quercetin have protective effect against oxidative stress and subsequent apoptosis in HUVEC cells.

## 1 INTRODUCTION

Cardiovascular diseases are known as the leading cause of global mortality (Mensah et al., 2019). Risk factors for cardiovascular diseases include hypertension, diabetes, low education, ambient air pollution, obesity, unhealthy diet, non‐high‐density lipoprotein (HDL) cholesterol, excess alcohol, and low physical activity (Yusuf et al., 2020). Oxidative stress plays a pivotal role in various human diseases and is a common feature in cardiovascular disease risk factors (Cammisotto et al., 2021). Oxidative stress refers to an imbalance between the production of oxygen‐reactive species (ROS) and the antioxidant defenses (Forouzanfar & Hosseinzadeh, 2020). Lipids, proteins, and DNA are the cellular biomolecules that can be harmed by oxidative stress (Siti et al., 2015). It is well established that oxidation of low‐density lipoprotein (LDL) particles contributes to the formation of oxidized LDL, which can be cytotoxic and cause the initial disruption of endothelial cells and subsequent injury to vascular walls (Siti et al., 2015; Tesfamariam & DeFelice, 2007). Previous studies showed several natural active substances had protective effect on vascular endothelial cells (Farshori et al., 2021; Guo et al., 2021; Liao et al., 2021). Numerous studies have shown that antioxidants originating from plants, such as vitamins E and C, tocopherols, β‐carotene, and polyphenols, may be protective against cardiovascular disorders (Siti et al., 2015; Wang et al., 2013). *Rosa canina* L., (*Nastaran* or *Nasrin* in Persian) a member of the Rosaceae family, is a thorny shrub with white flowers and bright red hips that has spread to several areas of the world. *R. canina* has been used in traditional medicine for hepatic illnesses, various neurological and gastrointestinal diseases, headaches, and as a tonic for the heart and brain (Taghizadeh et al., 2016). Phytochemical screening revealed that *R. canina* extracts contain active ingredients such as tannins, proanthocyanidins, flavonoids, phenolic acids, unsaturated and galactolipids, phospholipids, minerals, polyunsaturated fatty acids, and carotenoids (Chrubasik et al., 2008; Lattanzio et al., 2011). Studies show that the fruits of *R. canina* have antioxidant properties and inhibit free radicals (Orhan et al., 2009). A number of animal pharmacological studies confirm the effects of *R. canina* in reducing triglycerides and fasting sugar (Medina‐Leyte et al., 2020; Tang et al., 2020) and generally improving the risk factors of cardiovascular diseases (Taghizadeh et al., 2016). Quercetin (3,3′,4′,5,7‐pentahydroxyflavone) is a plant pigment compound that belongs to the flavonoids family. It has unique biological qualities such as an antioxidant, anticarcinogenic, anti‐inflammatory, neuroprotective, and antiviral; it can also suppress platelet aggregation, capillary permeability, and lipid peroxidation (Li et al., 2016; Tang et al., 2020). Quercetin is present in large amounts in *R. canina* (Chrubasik et al., 2008). According to the antioxidant effects of *R. canina* fruit and its components, the putative protective effects on oxidative damage to blood vessels are assumable. This investigation aims to examine the role of *R. canina* fruit extract (RCFE) and quercetin in preventing cell damage caused by H_2_O_2_ and to study the role of apoptosis. In this method, human umbilical vein endothelial cells (HUVEC) were used, which is an excellent model for investigating various aspects of cardiovascular and vascular function (Medina‐Leyte et al., 2020).

## 2 MATERIALS AND METHODS

### 2.1 Reagents

Propidium iodide (PI), 2′,7*′‐*dichlorofluorescein diacetate (DCF‐DA), complete protease inhibitor cocktail, resazurin, RPMI 1640, Tris‐buffered saline with Tween 20 (TBST), and H_2_O_2_ were purchased from Sigma; Ammonium persulfate (APS), PVDF membranes, dimethylsulfoxide (DMSO), tetramethylethylenediamine (TEMED), and other materials were purchased from Merck Millipore; and penicillin/streptomycin 100× and fetal bovine serum (FBS) were bought from Gibco. Anti‐β‐actin (13E5), PARP (9542), survivin (71G4B7), and horseradish peroxidase‐conjugated goat anti‐rabbit IgG (7074) antibodies were bought from Cell Signaling Technology.

### 2.2 Plant material and extraction method

Fruits of *R. canina* were collected from around Ardabil city in early autumn. Extraction was done by percolation method with 70% ethanol as follows. Three hundred grams of *R. canina* fruit powder was moistened with half a liter of solvent, and after one night, it was transferred to a suitable percolator and covered with an additional amount of solvent. After 24 h. The resulting extract was solvent removed by a rotary evaporator. After removing the solvent, the extract was transferred to a round flask and placed in the freezer for several days. Then, the balloon was connected to the freeze dryer and after about 14 days, it was separated and the extract was taken out.

### 2.3 Cell culture

HUVEC was purchased from the Cell Bank of the Pasteur Institute of Iran. HUVEC cells were cultured using a T75 cm^2^ flask in RPMI 1640 medium supplemented with 10% FBS, and 1% penicillin/streptomycin at a humidified 5% CO_2_ atmosphere at 37°C.

### 2.4 Cell viability

HUVECs were seeded at a density of 1 × 10^4^ cells/well per 96‐well plate. After 24 h, the medium was changed to medium containing the RCFE (1.25, 2.5, 5, 10, and 20 μg/mL) and quercetin (1.25, 2.5, 5, 10, and 20 μM). After 24 h of incubation, the HUVECs were exposed to H_2_O_2_ (1 and 2 mM for 60 min). After that AlamarBlue® was added to each well to each well, and the cells were incubated for an additional 4 h at 37°C. Next, the cell viability was determined by measuring the absorbance at 570 and 600 nm (background) using an ELISA microplate reader (Awareness; Tayarani‐Najaran et al., 2017).

### 2.5 Measurement of reactive oxygen species

HUVEC cells (10^4^ cell/well) were treated with the RCFE (1.25, 2.5, 5, 10, and 20 μg/mL) and quercetin (1.25, 2.5, 5, 10, and 20 μM) for 24 h. After 30 min exposure to different concentrations of H_2_O_2_ (1 and 2 mM), the cells were washed and loaded with 10 mM DCFH‐DA for 30 min at 37°C. The fluorescence intensity was measured at excitation wavelength: 485 nm and emission: 530 nm by microplate reader (Tayarani‐Najaran et al., 2021).

### 2.6 Determination of apoptosis

Apoptosis detection was performed with the PI staining. HUVEC cells (10^5^) were treated with the RCFE (2.5, 5 μg/mL) and quercetin (2.5, 5 μM). After 24 h treatment, cells were exposed to H_2_O_2_ (2 mM) for 60 min, and then, 400 μL of a hypotonic buffer containing 50 μg/mL PI in 0.1% triton X‐100 and 0.1% sodium citrate were added to each well after the cells had been harvested. Prior to flow cytometry analysis, the cells were cultured in the dark at 4°C for 30 min (FACS Scan, BD Biosciences; Tayarani‐Najaran et al., 2021).

### 2.7 Western blot analysis

After treating cells (10^6^) with 0, 2.5, and 5 μM quercetin and 0, 2.5, and 5 μg/mL RCFE for 24 h, the cells were centrifuged at 1500 rpm twice with cold PBS buffer, and the cell pellet was lysed in lysis buffer containing Tris 50 mM pH 7.4, complete protease inhibitor cocktail, 2 mM EDTA, 10 mM β‐glycerol‐phosphate, 10 mM NaF, 1 mM Na3VO4, 0.2% w/v sodium deoxycholate, and 1 mM PMSF. Cell lysate was collected after centrifugation at 10,000 rpm at 4°C for 20 min. Each protein sample that had been adjusted was loaded onto a 10% SDS‐PAGE before being transferred to a PVDF membrane. The membranes were incubated with the primary antibodies against surviving, PARP, and β‐actin for 2 h at 4°C after being blocked with 5% skimmed milk in 0.1% Tween 20 in PBS. The blots were washed three times for 10 min each with TBST, then incubated for 2 h at 37°C with the appropriate secondary antibodies (1:3000, v/v), and again washed with TBST (Rahiman et al., 2018). Enhanced chemiluminescence kit (ECL, Amersham Biosciences) was used to visualize the target proteins. Utilizing the Gel‐pro Analyzer V.6.0 Gel Analysis software, images were quantified (Media Cybernetics, Inc).

### 2.8 Statistical analysis

One‐way ANOVA followed by Tukey post hoc was performed to determine statistical significance test. All data are presented as mean ± SEM. *p* values less than .05 were considered statistically significant.

## 3 RESULTS

### 3.1 Effects of *R. canina* extract and quercetin on the viability of HUVECs

From 300 g of fruits, 90 g of extract was obtained. The percentage of the obtained extract was 30%. The 2 h exposure of HUVECs to H_2_O_2_ (1–2 mM) resulted in severe HUVEC loss compared to control group (Figure 1a,b). As illustrated in Figure 1a, RCFE (2.5, 5, 10, and 20 μg/mL) significantly attenuated HUVEC death induced by H_2_O_2_ (1 mM). Quercetin (1.25, 2.5, 5, 10, and 20 μM) significantly attenuated HUVEC death induced by H_2_O_2_ (1 mM). Concentrations of 2.5, 5, 10, and 20 μg/mL RCFE and concentrations of 5, 10, and 20 μM quercetin were able to significantly increase cell viability against 2 mM H_2_O_2_ (Figure 1b).

**FIGURE 1:** (a, b) Effects of the *Rosa canina* extract and quercetin on H_2_O_2_‐induced HUVEC cells' toxicity. The HUVECs pretreated with *R. canina* extract and quercetin for 24 h were exposed to 1 and 2 mM H_2_O_2_ for 30 min. *p < .05, ** *p* < .01, and *** *p* < .001 compared to H_2_O_2_. Values are the means ± SEM of three independent experiments.

### 3.2 Effects of *R. canina* extract and quercetin on H_2_O_2_ ‐induced ROS production in HUVECs

As shown in Figure 2a,b, a ROS burst was observed when cells were exposed to H_2_O_2_ (1–2 mM).

**FIGURE 2:** (a, b) Effects of the *Rosa canina* extract and quercetin on H_2_O_2_‐induced ROS generation in HUVEC cells. The HUVECs pretreated with *R. canina* extract and quercetin for 24 h were exposed to 1 and 2 mM H_2_O_2_ for 30 min. * *p* < .05, ** *p* < .01, and *** *p* < .001 compared to H_2_O_2_. Values are the means ± SEM of three independent experiments. R: *R. canina* extract, Q: quercetin.

Pretreatment of the cells with RCFE (5, 10, and 20 μg/mL) and quercetin (5, 10, and 20 μM) for 24 h significantly attenuated the elevation of ROS levels induced by H_2_O_2_ (1 mM).

Also, it was found that concentrations of 10 and 20 μg/mL of RCFE and 5, 10, and 20 μM of quercetin reduced the production of ROS by H_2_O_2_ in concentration of 2 mM.

### 3.3 Effects of *R. canina* extract and quercetin on H_2_O_2_ ‐induced apoptosis in HUVECs

As illustrated in Figure 3, the sub‐G1 peak (one of the reliable biochemical markers of apoptosis) in the flow cytometry histogram of H_2_O_2_‐exposed cells was greater than control cells (Figure 3). Treatment with RCFE (2.5 and 5 μg/mL) and quercetin (2.5 and 5 μM) could reduce the apoptosis rate.

**FIGURE 3:** Effects of the *Rosa canina* extract and quercetin on H_2_O_2_‐induced apoptosis in HUVEC cells. The HUVECs pretreated with *R. canina* extract and quercetin for 24 h were exposed to 2 mM H_2_O_2_ for 30 min. The test was performed in triplicate (*n* = 3). R: *R. canina* extract, Q: quercetin. 0.0: control.

### 3.4 Effects of *R. canina* extract and quercetin on the expression of apoptotic‐associated proteins

A significant reduction in the survivin level in H_2_O_2_‐exposed cells was observed, while RCFE (2.5 and 5 μg/mL) and quercetin (2.5 μM) protected against H_2_O_2_‐induced apoptosis in HUVEC cells (Figure 4a). Also, as shown in Figure 4b, the PARP level which is actually the first protein known as the substrate of caspases, increased significantly in H_2_O_2_‐exposed cells, while in the cells treated with RCFE (2.5 and 5 μg/mL) and quercetin (2.5 and 5 μM), the amount of PARP protein breakage significantly decreased against to the H_2_O_2_ group.

**FIGURE 4:** (a, b) Effects of the *Rosa canina* extract and quercetin on the amount of survivin and PARP proteins in H_2_O_2_‐treated HUVEC cells. β‐Actin was used as a protein‐loading control. The HUVECs pretreated with *R. canina* extract and quercetin for 24 h were exposed to 2 mM H_2_O_2_ for 30 min. ** *p* < .01, *** *p* < .001 compared to H_2_O_2_. Values are the means ± SEM of three independent experiments.

## 4 DISCUSSION

In the present study, we examined the protective effects of RCFE and quercetin, a flavonoid that exists in *R. canina* on HUVEC cells in the oxidative stress model induced by H_2_O_2_. The results showed that treating HUVEC cells with high concentrations of RCFE (5, 10, and 20 μg/mL) and quercetin (5, 10, and 20 μM) decreased H_2_O_2_‐induced cell damage and ROS production. The concentrations of 20 μg/mL of *R. canina* and 10 and 20 μM of quercetin showed better results in neutralizing free radicals. Given that the endothelium, which forms the inner cell lining of blood vessels and lymphatics, acts as an interface between components of the bloodstream such as monocytes and platelets and other components of the arterial wall, it is therefore vital in the development of cardiovascular diseases (Favero et al., 2014; Medina‐Leyte et al., 2020). HUVECs were first isolated from the umbilical cord and cultured successfully in 1973. To date, this model is still widely used because it is relatively easy to isolate, and HUVECs are useful to study a wide variety of diseases, including cardiovascular and metabolic diseases (Medina‐Leyte et al., 2020).

Another finding of this study was increase in the cell viability by inhibiting apoptosis following exposure to RCFE and quercetin. The protective properties were associated with changes in the survivin and PARP levels. Our study revealed that H_2_O_2_ could decrease survivin, while pretreatment with RCFE and quercetin increased survivin. Survivin, the smallest member of the inhibitor of apoptosis family of proteins, acts as a component of the chromosomal passenger complex, which plays an imperative role in the control of cell division (Li et al., 2018). Survivin is expressed during development and in proliferating adult cells (Wheatley & Altieri, 2019). PARP is a critical enzyme regulating a broad array of cellular functions, including modulation of chromatin structure, transcription, replication, recombination, and DNA damage repair. PARP binds to single‐stranded DNA and is important for repairing frequently occurring single‐strand breaks. The first protein to be inactivated by caspase 3 by enzymatic cleavage during the DNA damage process is PARP (Morales et al., 2014).

As expected from the previous reports, we here showed RCFE and quercetin protect both against the death induced by increase in ROS and apoptosis in HUVEC cells. The phenolic compounds and high‐vitamin C concentration in *R. canina* may be partially responsible for the plant's beneficial characteristics (Chrubasik et al., 2008). It has been confirmed in various researches that *R. canina* is able to reduce cardiovascular diseases by reducing blood pressure and LDL (Andersson et al., 2012; Selahvarzian et al., 2018). In addition to vitamin C, the fruit of the *R. canina* plant contains phytochemicals such as carotenoids, amino acids, tocopherol, tannins, pectin, sugars, bioflavonoids, organic acids, and essential oils. Also, *R. canina* fruit contains long‐chain unsaturated fatty acids, which are considered essential fatty acids, because the body cannot synthesize them. Linoleic and α‐linolenic acids are essential fatty acids whose health benefits include roles in the regulation of blood pressure, nerve function, membrane fluidity, blood viscosity, immune responses, inflammatory responses, and several other responses. The analysis of fatty acids showed that the main fatty acids in *R. canina* are composed of linoleic acid and α‐linolenic acid (Winther et al., 2016). In one study, by comparing the ability of *R. canina* fruit and five other fruits from the Rosaceae family to reduce hydroxyl radicals (OH) and hydrogen peroxide (H_2_O_2_), the total antioxidant activity of *R. canina* fruit was examined. The fruit's total phenol, ascorbic acid, and carotenoid concentrations were also evaluated. The phenolic and carotenoid content of *R. canina* was much higher than that of other analyzed fruits. The ascorbic acid level of *R. canina* fruit was also higher, which indicates its greater activity against H_2_O_2_ species (Egea et al., 2010). Also, aqueous extract of *R. canina* inhibits the chemotaxis of human peripheral blood leukocytes in laboratory conditions. These laboratory studies show that *R. canina* powder has anti‐inflammatory as well as antioxidant properties. Healthy and osteoarthritis individuals who consumed *R. canina* fruit powder every day for 4 weeks had reductions in polymorphonuclear leukocytes chemotaxis and levels of the inflammatory marker acute‐phase C‐reactive protein (CRP) (Kharazmi, 2008).

In humans, daily use of a *R. canina* fruit drink for 6 weeks (40 g/day), compared to the control drink, caused a significant decrease in systolic blood pressure, total plasma cholesterol, LDL, and LDL/HDL ratio. The Reynolds index for cardiovascular diseases was also reduced in osteoarthritis volunteers who received *R. canina* fruit compared to the control group. However, body weight, glucose tolerance, diastolic blood pressure, plasma levels of HDL, triglycerides, incretins, and inflammatory indices were not different between the two groups (Andersson et al., 2012).

In animals, blood pressure and oxidized LDL, atherosclerotic plaques, total cholesterol, and fibrinogen levels were significantly reduced in rats that received *R. canina* fruit, but it could not prevent weight gain or decreases in plasma glucose and insulin in ApoE‐null mice (Cavalera et al., 2017). In addition, administration of *R. canina* reduced the excessive production of ROS and inhibited the activity of caspase 8 caused by heat stress in the heart of male Wistar rats. Moreover, *R. canina* extract decreased the expression of p‐PERK, p‐eIF2α, and CHOP protein as heat stress‐related markers in endoplasmic reticulum of the heart (Nasrolahi et al., 2020). Quercetin, a potent antioxidant flavonoid that exists in *R. canina*, plays an imperative function in the prevention and treatment of atherosclerosis (Deng et al., 2020) (Chrubasik et al., 2008). Quercetin also effectively eliminates ROS and protects vascular endothelial function (Saw et al., 2014). One study showed that quercetin can protect endothelial function from oxidative stress induced by homocysteine by increasing the glutathione level, inhibiting protein oxidation, lipid peroxidation, and enzymatic reactions, and decreasing the malondialdehyde level in ‐homoc rats (Çelik et al., 2017). The results of the present study are in accordance with the antioxidant and anti‐apoptotic activity which were suggested in previous experimental and in vivo research.

## 5 CONCLUSION

This study shows that RCFE and quercetin protect HUVEC cells from H_2_O_2_‐induced cellular oxidative stress and apoptosis. Our findings demonstrate the therapeutic potential role of *R. canina* and quercetin in the treatment of cardiovascular illnesses. Consequently, further analytical and clinical research is warranted in order to strengthen the present findings.

## AUTHOR CONTRIBUTIONS

**Fatemeh Forouzanfar:** Supervision (equal); writing – original draft (equal). **Zeynab Tabatabaei:** Investigation (equal). **Seyed Ahmad Emami:** Supervision (equal). **Zahra Ayati:** Investigation (equal). **Zahra Tayarani‐Najaran:** Data curation (equal); supervision (equal).

## FUNDING INFORMATION

The work was supported by the Research Affairs of Mashhad University of Medical Sciences (Grant No. 971030).

## CONFLICT OF INTEREST STATEMENT

None.

## Data Availability

The data that support the findings of this study are available on request from the corresponding author.
